This article has been retracted.

# *PPP1*, a plant-specific regulator of transcription controls *Arabidopsis* development and *PIN* expression

**DOI:** 10.1038/srep32196

**Published:** 2016-08-24

**Authors:** René Benjamins, Elke Barbez, Martina Ortbauer, Inez Terpstra, Doris Lucyshyn, Jeanette Moulinier-Anzola, Muhammad Asaf Khan, Johannes Leitner, Nenad Malenica, Haroon Butt, Barbara Korbei, Ben Scheres, Jürgen Kleine-Vehn, Christian Luschnig

**Affiliations:** 1 Department of Applied Genetics and Cell Biology, University of Natural Resources and Life Sciences, Vienna (BOKU), Muthgasse 18, 1190 Wien, Austria; 2 Plant Developmental Biology, Wageningen University Research, 6708 PB Wageningen, The Netherlands; 3 Swammerdam Institute for Life Sciences, Faculty of Science, University of Amsterdam, 1090 GE Amsterdam, The Netherlands

## Abstract

Directional transport of auxin is essential for plant development, with *PIN* auxin transport proteins representing an integral part of the machinery that controls hormone distribution. However, unlike the rapidly emerging framework of molecular determinants regulating *PIN* protein abundance and subcellular localization, insights into mechanisms controlling *PIN* transcription are still limited. Here we describe *PIN2 PROMOTER BINDING PROTEIN 1* (*PPP1*), an evolutionary conserved plant-specific DNA binding protein that acts on transcription of *PIN* genes. Consistent with *PPP1* DNA-binding activity, *PPP1* reporter proteins are nuclear localized and analysis of *PPP1* null alleles and knockdown lines indicated a function as a positive regulator of *PIN* expression. Furthermore, we show that *ppp1* pleiotropic mutant phenotypes are partially reverted by *PIN* overexpression, and results are presented that underline a role of PPP1-*PIN* promoter interaction in *PIN* expression control. Collectively, our findings identify an elementary, thus far unknown, plant-specific DNA-binding protein required for post-embryonic plant development, in general, and correct expression of *PIN* genes, in particular.

The plant hormone auxin controls essential developmental processes throughout the life cycle of plants, which to a large extent depend on directional distribution of the growth regulator within the plant body^1^,^2^. Different families of membrane proteins mediating inter- and intracellular transport of auxin have been characterized, with *PIN* proteins involved in cellular efflux as well as in intracellular compartmentalization of auxin, and therefore subject to multifaceted control mechanisms^2^,^3^,^4^,^5^.

Next to post-translational regulation of *PIN* proteins, influencing direction and rates of polar auxin transport (PAT)^3^,^5^, there is accumulating evidence for a role of transcriptional control of *PIN* genes in the regulation of auxin distribution. This is indicated by observations linking adjustments in *PIN* transcript levels to various cues, such as environmental stimuli^6^,^7^,^8^ as well as plant growth regulators^9^,^10^,^11^. Furthermore, activity of several regulators of gene expression has been linked to *PIN* transcriptional control, thereby specifying morphogenetic processes in the course of plant development. This applies to members of the *PLETHORA* (*PLT*) family of transcription factors, activity of which has been associated with transcriptional regulation of *PIN* genes in the control of root morphogenesis^12^. A related scenario has been proposed for the regulation of meristem function, with protein complexes consisting of JAGGED LATERAL ORGANS (JLO), ASYMMETRIC LEAVES2 (AS2) and additional factors, shaping auxin distribution during organogenesis via *PIN* transcriptional control^13^. Moreover, members of the *INDETERMINATE DOMAIN* (*IDD*) family of transcription factors, implicated in diverse developmental processes, were found to be required for correct *PIN* transcription, pointing to an involvement in specifying auxin-controlled morphogenesis in plants^14^.

Evidence for a direct involvement in the transcriptional control of PINs has been provided for some regulatory proteins. *XAANTAL2/AGAMOUSLIKE14* (*XAL2/AGL14*), a MADS-box protein was found to associate with *PIN1* and *PIN4* loci, acting as a positive regulator of *PIN* expression in the control of root development^15^. Furthermore, analysis of *Arabidopsis* mutants deficient in BRAHMA (BRM) SWI2/SNF2 chromatin remodeling ATPase, revealed severe deficiencies in root stem cell niche maintenance, associated with a strong reduction in the expression of a subset of *PIN* genes^16^. Chromatin-IP (ChIP) experiments revealed BRM interaction with *PIN* loci, and genetic analysis positioned *BRM* and *PLT* genes in an overlapping pathway, apparently required for accurate control of auxin distribution via control of *PIN* expression^16^. Recently, control of *PIN* expression was found to depend on activity of *CYTOKININ RESPONSE FACTOR* (*CRF*) and *AUXIN RESPONSE FACTOR* (*ARF*) genes. ChIP assays demonstrated that members of each protein family associate with *PIN* gene promoter regions, evidently contributing to the transmission of hormonal signals in the regulation of *PIN* transcription^17^,^18^. Together, all these observations provide strong evidence for a scenario in which a stringent control of *PIN* transcription is essential for the regulation of PAT, and dynamics therein.

In this report, we describe another approach aiming at the identification of *PIN* transcriptional regulators by employing yeast one-hybrid (Y1H) methodology^19^. This led to characterization of *PIN2 PROMOTER BINDING PROTEIN1 (PPP1)*, an evolutionary conserved, plant-specific DNA-binding protein of unknown function. *In vitro* and *in vivo* evidence is provided, demonstrating *PPP1* interaction with *PIN* promoters, whereas a detailed *in planta* analysis identified *PPP1* as important transcriptional regulator of *PIN* genes as well as of PAT-controlled developmental processes. Altogether, our results define *PPP1* as founding member of a plant-specific family of DNA-binding proteins with an important role in transcriptional regulation of key determinants of plant morphogenesis and growth responses.

## Results

### Identification of a *PIN2* promoter interacting protein

A few regulators of gene expression have so far been demonstrated to influence *PIN* transcription via *PIN* promoter binding. In an attempt to identify further regulators we performed a Y1H screen, in which we used *PIN2* promoter fragments as baits that were fused to the baker’s yeast *HIS3* reporter gene^19^ (see Materials and Methods). The vast majority of analyzed candidate interacting proteins obtained from our screens, turned out to represent general DNA-binding proteins, such as histones as well as DNA modifying enzymes. In addition, when using a promoter fragment ranging from bp -1175 to bp -1002 with respect to the *PIN2* ATG start codon, we identified three independent cDNA clones, each corresponding to locus At5g08720. This suggested binding of the protein to the *PIN2* promoter fragment and therefore the corresponding gene was named *PIN2* PROMOTER BINDING PROTEIN 1 (*PPP1*).

A single ORF that encodes a predicted protein of approximately 82 kDa was identified in *PPP1* cDNAs. BLAST searches demonstrated that *PPP1* represents a single copy locus and structure/domain prediction (http://www.expasy.org/) resulted in identification of conserved motifs (Fig. 1a). *PPP1* contains two copies of a putative lipid-binding domain (aa 99-245 and aa 337-479), related to a domain found in members of the START superfamily (http://www.ncbi.nlm.nih.gov/Structure/cdd/cddsrv.cgi?uid=176942). This domain has been implicated in transport, binding and/or sensing of various hydrophobic compounds in pro- and eukaryotes^20^,^21^,^22^,^23^ Furthermore, we performed protein meta-structure analysis of *PPP1* by calculating residue compactness describing the structural complexity of an individual residue in the context of 3-D protein fold and local secondary structure elements^24^. This computational approach suggested a putative helix-turn-helix (HTH) structural motif, which extends from residue 575 to 615 (Fig. 1a; Supplemental Fig. 1), and could facilitate DNA-binding. In addition, we identified a potential bipartite Nuclear Localization Signal (NLS) in the very C-terminal portion of *PPP1* ranging from residue 664 to 697 that could signal nuclear localization of the protein (Fig. 1a; http://nls-mapper.iab.keio.ac.jp/cgi-bin/NLS_Mapper_form.cgi). No additional, characterized domains were predicted, but sequence entries related to *PPP1* were found in genomes of higher plants, fern and moss as well as of green algae belonging to the charophytes. In contrast *PPP1* orthologs were not found in the genomes of non-plant organisms, indicating that *PPP1* has evolved plant-specifically (Fig. 1b).

To verify *PPP1* interaction with the *PIN2* promoter we performed electrophoretic mobility shift assays (EMSAs) with purified, recombinant GST-tagged *PPP1* (GST-tPPP1), to test for DNA-binding of *PPP1 in vitro*. By using EMSA combined with deletion analysis, we first limited *PPP1*-binding to a promoter fragment of 40 nucleotides within the 176 bp *PIN2* fragment originally used in the yeast one-hybrid screen. Site-directed mutagenesis within this 40 bp fragment identified a DNA stretch of 16 bp as necessary for *PPP1*-binding *in vitro* (Fig. 1d), suggesting that *PPP1* associates with the *PIN2* promoter via this DNA domain. *In silico* analyses demonstrated that no further identical copies of the 16 bp motif can be found anywhere else in the *Arabidopsis* genome. Remarkably, when analyzing promoter regions of the additional *Arabidopsis PIN* genes, we identified a 5′ element of the *PIN2* sequence motif in the promoter regions of *PIN1*, *3*, *6*, *7* as well as *PIN8*, arguing for occurrence of partially conserved *PPP1* DNA-binding sites in the promoters of these *PIN* genes (Fig. 2a). When testing 33217 *Arabidopsis* promoter regions for the occurrence of the identified 7 bp DNA stretch we obtained 9430 hits in 8062 different loci, and we therefore wondered if appearance of this motif in 5 out of 8 *PIN* genes occurs just by coincidence. A hypergeometric test, in which we tested the probability to find this number of promoters or more with the 7 bp DNA stretch, given the total number of promoters with this 7-mer, indicated a significant enrichment of this 7 bp DNA stretch in *PIN* promoters (p < 0.024), which might reflect conservation of a DNA-binding motif involved in transcriptional control of *PIN* genes. (Fig. 2b).

*In silico* analyses provoked questions about the sequence specificity of *PPP1* DNA-binding *in vivo*, and we therefore analyzed *PPP1* in more detail, by using the Y1H system. Co-expression of *PPP1* fused to the GAL4 activation domain (AD-*PPP1*) together with *HIS3* under control of a minimal yeast promoter plus a *PIN2* promoter fragment (bp −1180 to bp −1004; Fig. 1c; AD-*PPP1*/*PIN*2p’::HIS) conferred growth on medium lacking histidine (Fig. 1c), whereas no efficient growth was detected in controls lacking *PPP1* (Fig. 1c; pACT/*PIN*2p’::HIS). We then used the *PIN1* promoter, containing a sequence motif related to the original *PPP1* DNA-binding site, as another bait in the Y1H system, which indeed gave rise to efficient yeast growth under selective conditions (Supplemental Fig. 1). Nevertheless, we also observed limited yeast growth when expressing AD-*PPP1* together with the *HIS3* marker gene under control of a yeast minimal promoter only (Fig. 1c; AD-*PPP1*/HIS3), and similar results were obtained for yeast *ADE2* when expressed by a minimal promoter (Supplemental Fig. 1). These findings are suggestive of limited DNA-binding specificity of *PPP1* when expressed in the heterologous host.

In further experiments, we asked whether or not *PPP1*, apart from DNA-binding, confers transcriptional auto-activation in yeast. To this end, *PPP1* was fused to the GAL4 DNA-binding domain to give BD-*PPP1*, which then was tested for its ability to activate GAL4-controlled reporter gene expression in yeast. In these experiments no significant *HIS3* reporter activation could be detected when expressing BD-*PPP1*, indicating that *PPP1* does not act as a transcriptional activator (Fig. 1c).

### In planta analysis of the *PPP1* DNA-binding domain

Our analysis of *PPP1* in yeast together with *in vitro* assays demonstrated DNA-binding activity of this plant-specific protein. In addition, our results argue for a restricted binding specificity of *PPP1*, but gave no conclusive insights into the role of *PPP1* DNA-binding *in planta*. To address this issue, we designed experiments, in which we tested for a requirement of the *PPP1* DNA-binding site for *PIN2* expression. We generated a *PIN2* translational reporter construct, in which the 16 bp stretch critical for *PPP1* binding *in vitro* was mutagenized (see Materials and Methods). The corresponding mutant *PIN2pm::PIN2:VENUS* and a wild type *PIN2p::PIN2:VENUS* construct were transformed into the agravitropic *eir1-4* (*pin2*) null allele and resulting transformants were analyzed for rescue of *eir1-4* root gravitropism defects, as this assay represents a reliable read-out for expression and functionality of the *PIN2* gene product^25^,^26^.

Among *eir1-4 PIN2p::PIN2:VENUS* control lines, 18% (n = 22 lines tested) exhibited subtle defects in root curling, but no obvious alterations in reporter expression. In addition, 9% (n = 22) showed agravitropic root growth, which coincided with a loss of *PIN2* reporter signals, possibly as a result of incorrect integration or silencing of the transgene. In *eir1-4 PIN2pm::PIN2:VENUS* lines we observed defects in root growth at a higher frequency, indicated by small aberrations in root waving when grown on the surface of solid medium inclined at an angle of 60° (53%; n = 38 lines tested; Supplemental Fig. 2). In addition, a fraction of the lines analyzed (21%; n = 38) exhibited strong root gravitropism defects (Supplemental Fig. 2). When analyzing *PIN2pm::PIN2:VENUS* expression in lines showing mild root growth aberrations, we infrequently detected subtle changes in reporter signal distribution, whereas *eir1-4 PIN2pm::PIN2:VENUS* lines with pronounced defects in root gravitropism exhibited distorted reporter expression, ranging from patchy signal distribution to a complete loss of reporter activity (compare Fig. 3a–c). This indicates that mutations in a *PIN2* promoter segment required for *PPP1*-binding *in vitro* impact on stable expression of the *PIN2:VENUS* reporter gene.

Spatiotemporal control of *PIN2* expression in root meristems was proposed to modulate auxin flow in response to environmental signals^25^,^27^. This model postulates that lateral *PIN2* expression gradients in gravistimulated roots, promote unequal auxin distribution to specify differential cell elongation in gravity-responding root tips^25^,^26^,^27^,^28^. In contrast, and unlike the situation in *eir1-4 PIN2p::PIN2:VENUS* root meristems (Fig. 3d), persistent *PIN*2 expression gradient formation was abolished in gravistimulated *eir1-4 PIN2pm::PIN2:VENUS*. Instead, we found irregular distribution of *PIN*2 reporter signals, frequently resulting in stochastic formation of *PIN*2 reporter signal gradients that appeared uncoupled from the direction of the gravity vector (Fig. 3e). Furthermore, we observed a relationship between *PIN2pm::PIN2:VENUS* reporter signal distribution and the orientation of root growth, with directionality of root growth towards the side of the root meristem that exhibited more intense *PIN*2 reporter expression (Fig. 3f,g; n = 15 roots; all exhibiting a reporter expression gradient in accordance with root bending). This is consistent with the idea that controlled variations in *PIN2* expression shape differential auxin distribution and tropic root growth and demonstrates that alterations in root gravitropism, associated with *eir1-4 PIN2pm::PIN2:VENUS*, coincide with deficiencies in *PIN2* expression control.

Overall our data illustrates that the identified *PPP1* binding site is required for the spatial and temporal gene activity of *PIN2* and its developmental role in gravitropism.

### *PPP1* is ubiquitously expressed and localizes to nucleus and cytoplasm

To study *PPP1* function *in planta* we first determined its expression. Data obtained from *Arabidopsis* arrays suggested expression of *PPP1* in a wide range of tissues and at different developmental stages (http://signal.salk.edu/cgi-bin/atta?CHROMOSOME=chr5&LOCATION=2843435). We performed whole mount *in situ* RNA hybridization experiments on young seedlings (2-3 DAG) and found *PPP1* expression in the root meristem, throughout cell division and elongation zones (Fig. 4a,b). Additional weaker signals were observed in the lateral root cap and in proximal layers of the columella root cap cells (Fig. 4a,b), indicating partial overlap with expression of the hypothetical *PPP1* target gene *PIN2* (Fig. 4c). Signals were also detected in true leaf primordia, further emphasizing *PPP1* expression in young, proliferative tissue (Fig. 4e). For additional analyses, we generated a transcriptional reporter, in which the β-glucuronidase (GUS) gene was expressed under control of a *PPP1* promoter fragment (see Materials and Methods). The corresponding *PPP1p::GUS* transgenic lines exhibited GUS-activity during vegetative and reproductive growth stages in a range of tissues, with signals most pronounced in vasculature and in proliferating tissue, including lateral root primordia and young leaves (Fig. 4d,f–h).

For sub-cellular localization studies we first aimed at translational fusions, with the Green Fluorescent Protein (GFP) expressed in frame with genomic *PPP1*, but when expressed *in planta* we failed to observe GFP signals sufficiently strong for further analysis, indicating limited abundance of the reporter protein. We therefore took another approach in which GFP was fused either to the 5′ or the 3′ end of the *PPP1* cDNA coding region and resulting fusions were expressed under control of the strong *35S*-promoter (*35S::GFP:PPP1* and *35S::PPP1:GFP*). Upon transient expression in onion epidermis cells, we detected nuclear localization and additional, weaker signals in the cytoplasm for both constructs (16 out of 18 cells for *35S::GFP:PPP1* and 11 out of 14 cells for *35S::PPP1:GFP*; Fig. 4i–k). A similar signal distribution was found in *Arabidopsis* lines, stably expressing either one of these reporter genes, characterized by prominent signals in nuclei of root meristem epidermis cells, together with weaker cytoplasmic signals (Fig. 4l-n; Supplemental Fig. 3). These results are suggestive of predominantly nuclear localization of *PPP1*, which would be consistent with a function in transcriptional regulation.

### *PPP1* is required for post-embryonic development and affects meristem activity

Next, we analyzed T-DNA insertion lines SALK_011411 (*ppp1-411*) and SAIL_175_B03 (*ppp1-476*), which contain insertions within the *PPP1* coding region, and found that both lines failed to produce adult homozygous progeny (Fig. 5a). Closer examination of segregating mutant populations resulted in identification of seedlings, which showed delayed development after 5 DAG and eventually arrested growth (Fig. 5b, Table 1). Genotyping of these lines confirmed that all growth-arrested seedlings tested were *ppp1-476/ppp1-476* and *ppp1-411/ppp1-411*, suggesting that a loss of *PPP1* interferes with post-embryonic development. Transformation of *PPP1/ppp1-476* plants with a wild type copy of *PPP1* complemented the mutant, giving rise to viable *ppp1-476/ppp1-476 gPPP1* T3 progeny, indistinguishable from wild type, and similar results were obtained when complementing *ppp1-411* (Supplemental Fig. 4). This indicates that severe growth deficiencies segregating in SALK_011411 and SAIL_175_B03 lines indeed result from a loss of *PPP1* function.

We observed defects in *ppp1* root morphology reflected in reduced meristem size and premature cell differentiation as well as aberrations in directional root growth (Fig. 5c–f). Lugol-staining of *ppp1* root meristems demonstrated a reduction in starch-accumulating columella root cap cells, and activity of *CYCB1*;*1*::*GUS* mitotic reporter was decreased in *ppp1* root meristems as well, emphasizing pronounced defects in root meristem activity and maintenance upon loss of *PPP1* (Fig. 5e–h). Assuming that *PIN* genes represent targets for *PPP1*, we analyzed expression of the auxin-responsive reporter gene *DR5::mRFP* in *ppp1* mutant root meristems^29^. These experiments revealed decreased reporter expression in the mutant (Fig. 5i,j), evidently reflecting alterations in auxin transport and/or signaling upon loss of *PPP1*.

### PPP1 modulates transcription of *PIN* genes

*In vitro* and *in vivo* evidence argues for a function of *PPP1* in the transcriptional regulation of gene expression, with *PIN* genes representing potential targets for the DNA-binding protein. Consistently, analysis of *PIN2::PIN2:VENUS* expression in *ppp1-476* root meristems demonstrated reduced reporter signals, when compared to segregating *PPP1* seedlings (Supplemental Fig. 5). Nevertheless, owing to the strong growth deficiencies associated with *ppp1* T-DNA insertion alleles, it appeared difficult to draw valid conclusions based on expression analysis performed with these mutants. We tried to overcome this limitation, and used an artificial microRNA approach for generation of leaky, less severe *ppp1* loss-of-function alleles^30^.

We obtained *35S*-promoter-driven *PPP1* amiRNA silencer lines (*ami-ppp1*) and expression analysis resulted in identification of transgenic lines, exhibiting down-regulation of *PPP1* transcription, but less pronounced than in *ppp1-411* (Fig. 6a, Supplemental Fig. 5). Moreover, these *ami-ppp1* lines turned out to resume growth beyond early development, and produced viable homozygous offspring, supporting the notion that *ami-ppp1* lines exhibit only a partial loss of *PPP1* function (Fig. 7c, Supplemental Fig. 5).

Next we tested transcription of *PIN* genes in *ppp1* loss-of-function lines. qPCR performed with *ppp1-411* did not allow for a reliable interpretation of gene expression, as transcript levels even of the marker genes used for standardization, exhibited strong fluctuations. This might have resulted from the severe growth defects associated with this mutant. Reproducible results were obtained when analyzing knock-down *ami-ppp1*, revealing a strong reduction in transcript levels of *PIN1* and *PIN2* (Fig. 6b). Consistently, when analyzing activity of the *PIN2p::GUS* reporter gene^31^, we detected reduced GUS-staining (Fig. 6c,d), and reduced *PIN*-specific signal intensity in whole-mount immunostainings performed with *ami-ppp1* seedlings (Fig. 6e,f). Overall, these findings indicate that *PPP1* is required for correct expression of *PIN* genes.

We also tested for effects of *PPP1* down-regulation on additional loci, implicated in inter- and intracellular auxin transport. Only moderate alterations were observed when assessing transcript levels of *PIN4*, *AUX1* and *LAX3* auxin uptake facilitators as well as *ABCB4*, an ABC-type transporter involved in auxin transport across the plasma membrane^32^,^33^,^34^,^35^ (Fig. 6g). Notably, none of these loci contains the 7-nucleotide motif, identified in some *PIN* promoters (Fig. 2), which might explain their limited response in *ami-ppp1*. Pronounced differences however, were observed when testing expression of some *PILS* genes, participating in the intracellular distribution of auxin^36^, with *PILS5* transcript levels reduced by more than 50%, whilst *PILS3* transcription exhibits a more than twofold up-regulation in *ami-ppp1* (Fig. 6g). We detected the 7-nucleotide consensus motif in the *PILS5* promoter (bp −426 to bp −432 with respect to its Start ATG), implying that reduced transcription could arise as a consequence of diminished *PPP1* binding to the *PILS5* promoter. On the contrary, neither *PIN3* nor *PIN7* exhibited altered transcription in *ami-ppp1*, despite the fact that promoters of both genes contain the 7-nunclotide consensus sequence (Fig. 2). Thus, whilst altered expression of only a subset of genes, tested in *ami-ppp1,* points to some degree of *PPP1* target site specificity, our results as well indicate that presence of this minimal consensus motif is not sufficient to confer distinct *PPP1* effects on gene expression.

Phenotypes associated with *ami-ppp1* lines are consistent with a function of *PPP1* in *PIN* transcriptional control. Similar to *ppp1* T-DNA insertion lines, *ami-ppp1* roots were shorter than wild type roots of identical age (Fig. 7a,b and d). Furthermore, *ami-ppp1* roots exhibited alterations in directional, gravitropic root growth, when grown on vertically positioned nutrient plates, a hallmark feature of mutants with defects in auxin transport and/or signaling^37^ (Fig. 7e, Supplemental Fig. 5). When analyzing aerial portions of *ami-ppp1* plants we observed a stunted growth phenotype, together with a delay in the development of inflorescences and siliques (Fig. 7c). Nevertheless, *ami-ppp1* transgenics turned out to be fertile and could be propagated as homozygous lines (Fig. 7d).

Reduced *PIN* transcript levels in *ppp1* loss-of-function lines, together with the observation that *PPP1* binds to *PIN* promoter fragments *in vitro* and/or *in vivo,* argue for a function of *PPP1* as a positive regulator of *PIN* genes. If true, then diminished *PIN* abundance should contribute to the phenotypes occurring upon loss of *PPP1*. We tested this hypothesis and crossed a *35S::PIN1* overexpression line into the *ppp1-411* allele. Resulting F3, homozygous for *ppp1-411* and *35S::PIN1* developed significantly longer primary roots than *ppp1-411* controls, also reflected in larger root meristems (Fig. 7f–h). Based on these observations we concluded that growth deficiencies associated with a loss of *PPP1* are to some extent attributable to reduced expression of *PIN* genes, and its consequences on directional auxin transport.

## Discussion

*PIN* proteins are controlled by a complex circuitry of protein sorting, protein localization and protein degradation events, which exert combinatorial effects on polar auxin transport^3^,^4^,^5^. *PIN* transcriptional regulation has been related to plant development as well^6^,^7^,^9^,^11^,^12^, and there is emerging information on regulatory proteins involved^15^,^16^,^17^,^18^. Here we introduce *PPP1,* a plant-specific DNA-binding protein that modulates *PIN* expression, plant development in general, and auxin responses in particular.

Defects in the regulation of *PIN* function have repeatedly been demonstrated to induce drastic aberrations in auxin-controlled processes, underlining a key function for *PIN*s throughout the lifecycle of plants. Apart from numerous studies addressing *PIN* sorting and distribution, further reports highlighted a critical role for spatiotemporal control of *PIN* dosage, which modulates diverse aspects of plant development. In contrast, mechanisms underlying *PIN* transcriptional control started to be revealed only very recently. This is somewhat surprising, since there is well-established experimental evidence indicating that variations in *PIN* transcription in response to environmental and intrinsic cues contribute to the implementation of developmental programs^6^,^7^,^8^,^9^,^10^,^11^. Furthermore, *PLT*-type transcription factors, representing essential regulators of plant development, have been implicated in *PIN* transcriptional control^12^, and another report highlighted a function of *ARABIDOPSIS RESPONSE REGULATOR 1* (*ARR1*) in the transmission of cytokinin signals on *PIN* transcription^38^. In mechanistic terms however, direct crosstalk between transcriptional regulators and *PIN* loci has not been demonstrated until very recently^17^,^18^.

*PPP1* belongs to a small group of proteins, so far demonstrated to associate with promoters of *PIN* genes, which makes it a likely regulator of *PIN* expression. However, unlike additional *PIN* promoter-interacting proteins characterized to date, which were demonstrated to bind to well-characterized conserved DNA binding motifs, no such motif has been identified for *PPP1*. *In silico* analyses led to identification of a 7-nucleotide sub-motif within the *PPP1* DNA-binding site from the *PIN2* promoter, which was found to be enriched in the promoter region of additional genes. Assuming that these motifs are recognized by *PPP1* as well, it might specify its role in transcriptional regulation. The outcome of our Y1H experiments and expression assays performed with *PIN1* and *PILS5*, both characterized by a copy of the 7-nucleotide motif in their promoters, is consistent with this hypothesis. In addition, transcript levels of additional loci, lacking this DNA motif, remained unaffected in *ami-ppp1*, pointing to a certain amount of specificity in *PPP1*-target site interaction. On the contrary, expression of *PIN3* and *PIN7*, which both contain the 7-nucleotide motif in their promoters, did not markedly respond to *PPP1* downregulation. Moreover, we observed *PPP1*-dependent activation of yeast reporter genes, expressed by minimal promoters lacking this motif, overall arguing for limited *PPP1* DNA-binding specificity. At this moment, we can only speculate about the biological significance of these observations, since *cis*-acting requirements for *PPP1* DNA-binding and transcriptional control are not entirely explained. For example, it cannot be excluded that additional components, absent in yeast and *in vitro* experiments, confer specificity to *PPP1*-DNA interactions. Protein-protein interaction and complex formation have been demonstrated to define DNA binding activities, crucial for the transcriptional regulation of a wide range of target genes^39^,^40^,^41^. By analogy, identification of *PPP1*-interacting factors, together with a genome-wide documentation of *PPP1* DNA-binding sites should enable an in-depth characterization of binding specificities and activities of this so far unknown DNA-binding protein.

Indirect evidence for a requirement of *PPP1* in the regulation of *PIN2* transcription comes from analysis of *PIN2mp::PIN2:VENUS*, mutagenized in its *PPP1 in vitro* binding site. Although only incomplete conservation of DNA motifs appears to be required for *PPP1* binding, mutations within this *PIN2* promoter fragment resulted in stochastic variations or even a total loss of gene expression, at a frequency considerably higher than in controls. This suggests that the *PPP1* binding site in the *PIN2* promoter is essential for specifying or maintaining the expression status of the reporter gene *in vivo*. The extensive variability in VENUS signals observed in the different *eir1-4 PIN2mp::PIN2:VENUS* lines would be consistent with a general function of *PPP1*, ensuring stable expression of *PIN2* and presumably a range of additional loci, including further auxin transport proteins such as *PIN1*. A related model has been put forward for *Arabidopsis* BRM chromatin remodeling ATPase, with a rather broad spectrum of targets, amongst which expression control of *PIN* genes appears to play a key role^16^. In fact, a loss of *BRM* was found to cause reduced expression of *PIN* genes, together with severe developmental aberrations, resembling defects associated with *ppp1* loss-of-function lines. Notably, patchy *PIN*2-VENUS signals that we observed are a characteristic feature of reporter genes that underwent somatic gene silencing events. This might argue for an involvement of the *PPP1* DNA-binding motif in controlling the epigenetic status of the *PIN2* promoter region. If true, then chromatin association of *PPP1* could have an active function in transmission or maintenance of epigenetic signatures required for the correct expression of target genes, analogous to *BRM*. Clearly, genome-wide identification of *PPP1* targets, together with an in-depth analysis of *ppp1* loss-of-function lines will aid the analysis of *PPP1* and its role in the regulation of gene expression.

Phenotypes that co-segregated with two distinct T-DNA insertion lines disrupted in *PPP1*, demonstrated an essential role for the corresponding gene product. However, the factual growth arrest, occurring a few days after germination, makes these *ppp1* alleles rather inaccessible to an instructive phenotypic characterization. Analysis of *ami-ppp1* plants on the other hand, established a link to the control of auxin-dependent growth and development. This is emphasized by *ami-ppp1* growth defects, resembling phenotypes of auxin-related mutants as well as by a reduction of *PIN1* and *PIN2* transcript levels, which is consistent with *PPP1* modulating auxin distribution via transcriptional control of *PIN* genes. Conversely, the strong phenotypes of the likely *ppp1* null alleles do not necessarily reveal connections to auxin signaling. Limited DNA-binding specificity, which is indicated by our experiments, suggests a broader range of *PPP1* targets, presumably affecting expression of *Arabidopsis* loci unrelated to auxin transport or signaling, which offers a straightforward explanation for the severe defects associated with the *ppp1* knockout alleles. Partial rescue of *ppp1-411* root growth defects caused by constitutive overexpression of *PIN1* however, is in agreement with a function of *PPP1* as a fundamental, positive regulator of *PIN* genes, shaping intercellular auxin distribution and plant development.

When assuming a broad range of *PPP1* targets, distinct phenotypes of leaky *ami-ppp1* alleles, reflecting aberrations in auxin-related processes, appear unexpected to some extent. Similar observations have been made upon interference with basic cellular processes, such as endocytic sorting or translational control, disturbance of which repeatedly resulted in auxin-related growth defects^42^,^43^,^44^. Such observations led to models in which auxin signaling exerts rate-limiting functions during plant development, manifested as defined auxin-related growth aberrations even upon disturbance of highly general cellular mechanisms. A similar scenario could be envisioned for *PPP1,* acting as a pleiotropic regulator in plant development, with its function as a positive regulator of *PIN* transcription contributing to distinct aspects of auxin-controlled morphogenesis.

At present we can only speculate about mechanisms by which *PPP1* might influence gene expression. Circumstantial evidence for a role of *PPP1* as part of regulatory protein interaction networks comes from work published in recent years^45^,^46^. Dortay and colleagues demonstrated *PPP1* interaction with type-A ARABIDOPSIS RESPONSE REGULATORS (ARR), which act as repressors of transcriptional responses in cytokinin signaling^46^,^47^. Stegmann and coworkers on the other hand, demonstrated interaction between *PPP1* and plant U-box–type E3 ubiquitin ligase PUB22 that is essential for pathogen-associated molecular pattern-(PAMP)-triggered responses in *Arabidopsis*^45^. Although the biological significance of these protein interactions remains to be determined, it establishes links to environmental and hormonal control of plant development. In this context, it is worthwhile noting that *PPP1* contains two START-domains that form structurally conserved cavities predicted to interact with hydrophobic binding partners^48^. Furthermore, this domain has been identified in a family of plant receptor proteins, where it was found to be indispensable for binding of the phytohormone abscisic acid^49^. Although possible ligands recognized by *PPP1* are currently not known, it is tempting to speculate about a role for *PPP1*-ligand interaction with respect to its function in transcriptional regulation. Studies that will characterize *PPP1* START-domains and its interaction partners should help to obtain insights into the function of this plant-specific DNA-binding protein.

## Methods

### One-hybrid screens and yeast experiments

The yeast one-hybrid system described in Ouwerkerk and Meijer (2001) was used to screen an *Arabidopsis* cDNA library fused to the GAL4-activation domain (pACT2)^19^,^50^. A set of *PIN2* promoter restriction enzyme-cut fragments has been employed for identification of promoter binding proteins, namely EcoRV (nt. -2159) - BglII (nt. -1685); BglII (nt. -1685) - BalI (nt. -1429); BalI (nt. -1429) - NruI (nt. -1175); NruI (nt. -1175) - PmlI (nt. -1002); PmlI (nt. -1002) - BamHI (nt. -572); BamHI (nt. -572) - XbaI (nt. -329). *PPP1* cDNA clones were obtained, when using the PmlI (nt. -1002) – NruI (nt. -1175) *PIN2* promoter fragment as bait cloned into pINT1^19^ (pINT1-PIN2p’-HIS3) for transformation into yeast strain Y187 (Clontech). We transformed this strain with the pACT2 library DNA using standard conditions and screened for growth in the absence of histidine^50^. Approximately 2 × 10^6^ yeast transformants were screened both at RT and at 30 °C. For transactivation analysis the *PPP1* cDNA was cloned into pGBKT7 (Clontech), and expressed in yeast strain PJ69-4A^51^. A fragment covering 2.0 kb of the *PIN1* promoter region was cloned into pMW#2 using Gateway cloning^52^ (Invitrogen, Carlsbad, USA). Interaction of these with *PPP1* was tested in strain YM4271 on SC medium, lacking histidine and leucine and complemented with 20 mM 3-AT.

### Protein production and EMSA

For electrophoretic mobility shift assays (EMSAs) an EcoRI-XhoI *PPP1* fragment was cloned into pGEX4T-2, expressing a truncated version of *PPP1* ranging from amino acid residue 113 to 642. *E. coli* BL21-DE3 cells were used for heterologous expression of the recombinant protein. GST:tPPP1 was purified by binding to a gluthathione-sepharose matrix (Fluka/Sigma-Aldrich, St. Louis, USA) essentially as described^43^. Purified recombinant protein was used in EMSAs using end-labeled *PIN2* promoter fragments as described^53^. Binding assay reactions contained 4 μl of 5× binding buffer (0.25 M KCl; 25 mM MgCl2; 0.1 M Tris-HCl (pH8.0); 30% glycerol); 2 μl polydIdC (1 mg/ml); 1 ng end-labelled DNA-probe (1 ng/μl), GST-tPPP1 (app. 2–20 ng), and water to a final volume of 20 μl. EMSAs were performed at least two times.

### Plant materials and transgenic lines

Plants were grown on plant nutrient agar plates (5 mM KNO_3_, 2 mM MgSO_4_, 2 mM Ca(NO_3_)_2_, 250 mM KPO_4_, 70 μM H_3_BO_3_, 14 μM MnCl_2_, 500 nM CuSO_4_, 1 μM ZnSO_4_, 200 nM Na_2_MoO_4_, 10 μM NaCl, 10 nM CoCl_2_, 50 μM FeSO_4_; pH adjusted to 5.7; supplemented with 1% (w/v) agar and 1% (w/v) sucrose^54^ in 16 hrs light/8 hrs dark regime at 21 °C. *PIN2p::GUS*, *DR5::mRFP*, *35S::PIN1* and *eir1-4* (SALK_091142) have been described previously^25^,^29^,^31^,^55^. A *PPP1* artificial microRNA construct was designed using the web tool on the website of the Weigel laboratory by using oligonucleotides I-ppp1-ami 5′-GATATGTCATAACGACCTGCTGGTCTCTCTTTTGTATTCC-3′; II-ppp1-ami 5′-GACCAGCAGGTCGTTATGACATATCAAAGAGAATCAATGA-3′; III-ppp1-ami 5′-GACCCGCAGGTCGTTTTGACATTTCACAGGTCGTGATATG-3′; IV-ppp1-ami 5′-GAAATGTCAAAACGACCTGCGGGTCTACATATATATTCCT-3′ (weigelworld.org)^30^. The ami-RNA construct was subsequently cloned under control of the 35S-promoter into the binary pGREENII-0125 vector, with its resistance cassette replaced by a Norflurazon resistance marker (gift from Renze Heidstra, Wageningen University), using Gateway. All plant transformations were performed using the floral dip method^56^ and the Col-0 ecotype, if not indicated otherwise. *PPP1p::GUS* was generated by PCR amplification of a *PPP1* promoter fragment ranging from nt. -1112 to nt. -1 relative to the predicted *PPP1* start ATG by using primers 5′-AAGTCGACTTCTACCGTTGAATTCTCACAGAT-3′ and 5′-AAGTCGACTAGCGAAAGGTGTTCGACGAA-3′. The resulting fragment was cloned into pPZP-GUS^57^. The vectors for bombardment of onion epidermal cells (for method see below) were generated using Gateway. For generating the C-terminal GFP fusion to *PPP1*, driven by the 35S-promoter, the *PPP1* cDNA lacking the stop codon was amplified using the oligonucleotides 5′-GGGGACAAGTTTGTACAAAAAAGCAGGCTTTATGTCAGTGAGCAAGTTTCCACATCTC-3′ and 5′-GGGGACCACTTTGTACAAGAAAGCTGGGTCATATTGAACCCAATTGATATCAAGATCTTT-3′. The amplified PCR fragment was recombined by a BP reaction into pGEM-Teasy containing the Gateway recombination sites, creating pGEM-Teasy-*PPP1* min. pGEM-Teasy-*PPP1* min was subsequently used in a LR reaction with the destination vector pK7FWG2, thus creating pK7FWG2-*PPP1* min. For generating the N-terminal GFP fusion driven by the 35S-promoter, the *PPP1* cDNA lacking its start codon and containing the stop codon was amplified using oligonucleotides 5′-GGGGACAAGTTTGTACAAAAAAGCAGGCTTTTCAGTGAGCAAGTTTCCACATCTCTCT-3′ and 5′-GGGGACCACTTTGTACAAGAAAGCTGGGTCTCAATATTGAACCCAATTGATATCAAGATCT-3′. The amplified PCR fragment was recombined by a BP reaction into pGEM-Teasy containing the Gateway recombination sites, creating pGEM-Teasy-*PPP1*plus. pGEM-Teasy-*PPP1*plus was subsequently used in a LR reaction with the destination vector pK7WGF2. For generation of *PIN2pm::PIN2:VENUS* we performed site directed mutagenesis on *PINp::PIN2:VENUS*^26^ by using primers 5′-TCGCGATGATCGTGTAGATTTTTTTTTTTTTTTTGAATTGATGG-3′ and 5′-CCATCAATTCAAAAAAAAAAAAAAAATCTACACGATCATCGCGA-3′. After confirmation by sequencing, the construct was transformed into *eir1-4*. T2 pools of randomly picked primary transformants were analyzed for fluorescent signals on a Leica binocular and a Leica SP5 Confocal Laser Scanning Microscope (CLSM). In total, we screened 38 *eir1-4 PIN2pm::PIN2:VENUS* T2 populations that exhibited a 3:1 segregation for the transgene. Root growth responses were determined on seedlings germinated on vertically oriented nutrient plates. For *ami-ppp1* lines, 1.5% agar plates were used at an inclined angle of 60°, as these conditions make the *ami-ppp1* root phenotype more apparent.

The *ppp1* T-DNA insertion alleles SALK_011411 (*ppp1-411*) and SAIL_175_B03 (*ppp1-476*), were from the Nottingham Arabidopsis Stock Centre (NASC, www.arabidopsis.info) and genotyped by using oligonucleotides 5′-CCACCCATTCTTGTAATGGC-3′, 5′-GCATGAGATTCGTGAGCAG-3′ for *ppp1-411* and 5′-CCTAAGTAACCAATGCAATGAGTGCA-3′, 5′-GAATGTTCTTACTGATTATGAACGA-5′ for *ppp1-476*. For complementation we introduced a genomic T-DNA cosmid clone harboring the entire *PPP1* locus into *PPP1/ppp1-476* plants^58^. T3 progeny homozygous for the T-DNA clone was subsequently scored for homozygosity of the *ppp1* mutation. A similar setup was used for complementation analysis of *ppp1-411,* but a *PPP1p::cPPP1* T-DNA construct was used instead. *DR5-mRFP*, *CYCB1;1:GUS* and *PIN2p::PIN2:VENUS* were introduced into *ppp1-476* by crossing with heterozygote *PPP1/ppp1-476*. Analysis was performed in F2 and F3 generations.

### *In situ* mRNA hybridization and immunofluorescence

For whole-mount *in situ* hybridization^59^ a gene-specific 277-bp *PPP1* cDNA fragment ranging from nucleotide 1711 to 1989 was used for probe synthesis. The fragment was amplified and subsequently cloned into pGEM-T Easy (Promega). Subsequently, T7- and SP6-specific primers were used to synthesize anti-sense and sense probe, respectively.

Whole-mount immunofluorescence was performed as described^43^. Antibodies were diluted as follows: 1:500 for rabbit anti-PIN1^27^, anti-PIN2^25^ and 1:300 for FITC-conjugated anti-rabbit secondary antibodies (Dianova).

### Microscopy and staining procedures

Standard conditions were used for GUS staining with adaptation of concentrations for potassium ferricyanide and potassium ferrocyanide in the staining buffer (0.2 and 0.5 mM)^31^. Pictures of GUS-stained plant material were generated on a Zeiss Axio Imager A1 microscope, equipped with a CCD camera, using DIC-settings. Propidium iodide staining of seedlings was performed using a 10 μg/ml dilution in water for 2–5 minutes. CLSM pictures were generated by using a Zeiss Axio Imager M2 confocal microscope with 488 nm excitation and 495–565 nm emission for GFP, 514 nm excitation and 521–592 nm for VENUS, and 541 nm excitation with 575–620 nm emission for mRFP. For quantification of DR5::mRFP signals ImageJ software was employed.

### Transient expression in onion cells

5 μg of DNA were delivered into onion epidermal cells using gold particle bombardment. Gold particles (1.0 μm; Bio-Rad, Hercules, CA, USA) were coated with DNA according to the manufacturer’s directions. Particles were bombarded into onion epidermal cells using a Biolistic PDS-1000/He system (Bio-Rad) with 1100 psi rupture discs under a vacuum of 28 inHg. After bombardment, the cells were allowed to recover for 16–24 h on agar plates at 22 °C in the dark, after which positive cells were identified using a Leica MZ16F UV-binocular equipped with a GFP filter set. Subsequently, GFP positive cells were analyzed with a Zeiss Axio Imager M2 confocal microscope using 488 nm excitation and 495–565 nm emission wavelengths.

### RNA isolation and qRT-PCR

Whole RNA of seedlings (5 DAG) was extracted using the innuprep Plant RNA kit (Analytik Jena) from which cDNA was synthesized using the iScript cDNA synthesis kit (Biorad). qRT-PCR analysis was performed using a Biorad CFX96 Real time system with the IQ SYBRgreen super mix (Biorad) according to manufacturers’ recommendations. qRT-PCR was carried out in 96-well optical reaction plates heated for 3 minutes to 95 °C to activate hot start Taq DNA polymerase, followed by 40 cycles of denaturation for 10 seconds at 95 °C, annealing for 30 seconds at 55 °C and extension for 30 seconds at 72 °C. Expression levels were normalized to the expression levels of 2 household genes (*EIF4a* and *TUB*) using the Livak method^60^. Each experiment has been carried out with at least 3 biological replicates in 4 technical repetitions. Oligonucleotides that have been used for qPCR are listed in Supplementary Table S1.

### Domain prediction

In brief, the calculation of meta-structural parameters is based on statistical distributions of 3D atomic coordinates extracted from the Protein Data Bank (PDB) database (http://www.wwpdb.org/). From the 3D coordinate files, distances between amino acids A and B were extracted and scored as a function of amino acid types (A, B). Additionally, the primary sequence distance between residues A and B was taken into account. To describe the spatial neighborhood of the two amino acids in the 3D structure of the entire protein (e.g. the way the two amino acids are embedded in the 3D fold), the pairwise distance distributions were transformed from cartesian space (distance rAB) to topological space (dAB). dAB reflects differential structural neighborhood properties of two amino acids (A,B) and can be used to predict topological information (compactness parameter) and local secondary structure elements. Further information is provided in Konrat (2009)^24^. The compactness value is related to local residue exposure. Residues located in stable parts or in the interior of the protein structure have large values, whereas flexible loop regions and residues exposed to the solvent show small values. The average residue compactness value of stably folded proteins is about 300. Local secondary structure values range from −300 to +300. α–helices display positive values, β-strands show negative values.

### Phylogenetic analysis and DNA binding site predictions

For phylogenetic analysis we used the following sequence accessions compiled at Pubmed, MIPS, and JGI: *M. truncatula*, ABE86175; *O. sativa*, BAF13748; *P. patens*, XM_001783694; *V. vinifera*, XP_002273364; *O. tauri*, XP_003074385; *O. lucimarinus*, XP_001415547; *S. bicolor*, XP_002466133; *R. communis*, XP_002522916; *P. trichocarpa*, XP_002307063; *S. lycopersicum*, gene:scaffold00395_179.1; *Chlorella sp.* NC64A, ChlNC64A_1|57236|estExt_fgenesh3_pg.C_50136; *M. guttatus*, mgv1a002542m; *C. papaya*, supercontig 37.46; *C. sativus*, *Cucsa* 357500; *G. max*, Glyma04g38450, Glyma05g32950, Glyma06g16600, Glyma08g00580; *S. moellendorfi*, Selmo1|117904|e_gw1.57.486.1; *B. distachyon*, Bradi1g02450.2; *A. lyrata*, XP_002873379; *A. thaliana*, NP_680157. Multiple sequence alignments were performed with ClustalX by using default settings^61^. The resulting alignment was used for generation of a neighborhood-joining tree, corrected for multiple substitutions in the alignment and an exclusion of gapped positions. Statistical support for branches was calculated with bootstrap replicas (n = 100).

For the *in silico* analyses the genome sequence was obtained from the Bioconductor annotation package BSgenome.Athaliana.TAIR.TAIR9^62^. Motif occurrence in the genome was determined in R using the BioStrings package^63^. The promoter sequences 3000 kb upstream of the transcription start site were obtained from the Bioconductor annotation package TxDb.Athaliana.BioMart.plantsmart25^64^. Using pairwise alignment the 16-bp promoter fragment was aligned to the *PIN* promoters. With package SeqLogo^65^ the sequence logo of the aligned promoter regions was created. The 7 bp DNA fragment was matched against promoter sequences. The hypergeometric test was performed to assess the significance of enrichment of the 7-mer in a subset of the promoter sequences.

## Additional Information

**How to cite this article**: Benjamins, R. *et al*. *PPP1*, a plant-specific regulator of transcription controls Arabidopsis development and *PIN* expression. *Sci. Rep.* **6**, 32196; doi: 10.1038/srep32196 (2016).

## Supplementary Material

Supplementary Information

## Figures and Tables

**Figure 1:** Characterization of *PPP1* as DNA-binding protein. (**a**) Conserved domains predicted in the *PPP1* ORF (START domain, orange; putative HTH-motif, blue; bipartite NLS, yellow). (**b**) Phylogenetic relations of full-length *PPP1* and inferred *PPP1*-related protein coding sequences. Bootstrap support equal/greater than 50% is indicated on nodes and branch lengths are proportional to the number of substitutions per site (see scale bar). (**c**) Analysis of *PPP1* by Y-1-H. The yeast *HIS3* gene under control of either a minimal promoter (“HIS3”) or fused to a *PIN2* promoter fragment (“PIN2p’::HIS”) was co-expressed with *PPP1* fused to the GAL4 activation domain (“AD-*PPP1*”). Dilution series of these yeast cells were plated on complete SC medium (SC+His) and on SC lacking histidine supplemented with 10 mM 3-AT (SC-His/3-AT). Controls were performed with the *GAL4* activation domain only (“pACT”). For assaying transactivation activity, *PPP1* was fused to the *GAL4* DNA binding domain (“BD-*PPP1*”) and co-expressed with the *HIS3* gene under control of a *GAL* promoter (“GAL-HIS3”). Dilution series of yeast cells were spotted onto SC+His and on SC lacking histidine (asterisk: no 3-AT added to the medium). Growth was scored after 5 days incubation at 23 °C. (**d**) EMSA performed with GST:tPPP1 and a labeled 40 bp *PIN2* promoter fragment (*PIN2-BD*; nt. –1180 to nt. –1140 with respect to the predicted *PIN2* start ATG). Top: DNA sequences of wild type competitor (“comp.”) and mutant *PIN2* promoter fragments (“mut. comp.”) used for EMSA displayed below. Residues that have been exchanged are highlighted in red. Bottom: EMSA performed with GST:tPPP1. GST:tPPP1/PIN2-DB nucleoprotein complexes are indicated by arrowheads. No shift was observed in the absence of GST:tPPP1 (leftmost lanes) or, when using GST instead of GST:tPPP1 (“GST”). For the binding competition experiments we used 1x, 2x, 4x, 10x, 25x, 50x and 200x (from left to right) concentrations of unlabeled competitor DNA.

**Figure 2:** *In silico* analysis of *PPP1* DNA-binding sites. (**a)** Alignment of *PIN* promoter fragments. Nucleotides identical to the 16 bp motif characterized in the *PIN2* promoter are in red. A 7-nucleotide motif found in the promoters of *PIN1*, *PIN2*, *PIN3*, *PIN7* and *PIN8* is highlighted in yellow. Sequence logo displaying the position frequency matrix of aligned sequences of *PIN1*, *PIN2*, *PIN3*, *PIN6*, *PIN7* and *PIN8*. (**b)** Plot of all 16384 possible 7-mers matched to the promoter regions of 33217 *Arabidopsis* genes (x-axis), and to the promoters of all 8 *Arabidopsis PIN* genes (y-axis). For each 7-mer, a p-value is calculated based on the hypergeometric distribution, with hits with a p-value < 0.05 shown in black. The minimum 7-nucleotide common sequence found in the *PIN* promoters is depicted in red and circled.

**Figure 3:** Analysis of a predicted *PPP1* DNA-binding site *in planta*. (**a**) *PIN2p::PIN2:VENUS* expression in *eir1-4* root meristem epidermis cells at 4 DAG. (**b,c**) *PIN2pm::PIN2:VENUS* signals in root meristems in the progeny of two transformed lines at 4 DAG: Limited (b) and pronounced (c) alterations in reporter expression are indicated by arrowheads. (**d**) *PIN2p::PIN2:VENUS* expression gradient after 90 minutes of gravistimulation in a primary root meristem at 4 DAG (red arrowhead: direction of gravity vector; white arrowheads indicate differential PIN2-VENUS abundance). (**e**) Lateral *PIN2pm::PIN2:VENUS* expression gradient in a vertically oriented seedling at 4 DAG (red arrowhead: direction of gravity vector; white arrowheads indicate differential PIN2-VENUS abundance). (**f**) *eir1-4 PIN2pm::PIN2:VENUS* seedling at 7 DAG grown on a vertically oriented nutrient plate (red arrowhead: direction of gravity vector). (**g**) Higher magnification of the seedling’s root tip depicted in F (white rectangle). White arrowheads indicate VENUS signal gradient. Bars: a–e = 50 μm; f = 1 mm; g = 75 μm.

**Figure 4:** Expression analysis of *PPP1.* (**a,b**) Root whole-mount *in situ* RNA hybridization at 3 DAG performed with *PPP1*-specific antisense (a) and sense (b) probes. (**c**) *PIN2p::GUS* expression in the primary root meristem (5 DAG). (**d**) *PPP1p::GUS* activity in a flower (32 DAG). (**e**) Apical portion of wild type seedling (3 DAG) probed with *PPP1* antisense transcript (arrowheads indicate leaf primordia). (**f–h**) *PPP1p::GUS* activity in a lateral root primordium (10 DAG; f), in the shoot apical meristem region of a seedling (7 DAG; g), in the vasculature of a true leaf (20 DAG; h). (**i–k**) *PPP1*:GFP (i), GFP:*PPP1* (j) and nuclear-localized JKD:GFP^66^ (k) in onion epidermis cells (white arrowheads indicate cytoplasmic signals, red signals indicate PI-stained cell walls). **l**) Root stem cell niche showing *35S::PPP1:GFP* expression in nuclei and cytoplasm. (**m,n**) Details on *35S::PPP1:GFP* localization in reporter lines exhibiting strong (m) or weaker reporter expression (n). Green signals indicate reporter protein localization in nucleus and cytoplasm. Bars: a–c, e–g = 50 μm; d,h = 1 mm; i–k = 100 μm; l = 25 μm; m = 10 μm; n = 20 μm.

**Figure 5:** Analysis of *ppp1* loss-of-function alleles. (**a**) Position of T-DNA insertions in the genomic *PPP1* locus. (**b**) Wild type (left), *ppp1-411* (middle) and *ppp1-476* (right) plantlets at 16 DAG. (**c,d**) Primary roots of wild type (c) and *ppp1-411* at 10 DAG (d) grown on vertically oriented plates. (**e,f**) Lugol-staining of wild type (e) and *ppp1-411* (f) root meristems at 14 DAG. White arrowhead indicates onset of cell expansion. (**g,h**) Activity of *CYCB1;1::GUS* in wild type (g) and *ppp1-476* (h) root meristems at 10 DAG. (**i)** Expression intensities of *DR5::mRFP* in wild type (i) and *ppp1-476* (j) root meristems. (j) Quantification of *DR5::mRFP* signal intensities in the 1^st^ and 3^rd^ layer of root cap columella cells at 6 DAG (root cap cells from ≥10 seedlings were analyzed for each genotype; statistical analysis was performed using Student’s two-tailed t-test; error bars indicate standard deviations. Bars: b = 10 mm; c,d = 1 mm; e,f = 20 μm; g,h = 50 μm; i = 10 μm.

**Figure 6:** Expression profiling upon loss of *PPP1*. (**a**) qPCR analysis of *PPP1* expression in wild type (“WT”) seedlings versus *ppp1-411* insertion mutant seedlings (left) and an *ami-ppp1* silencer used for further analysis (right; see text). Graphs depict expression fold change in *PPP1* expression in *ppp1-411* and *ami-ppp1* relative to WT and normalized to the expression of 2 reference genes (*EIF4a* and *TUB*). Error bars depict s.e.m. from 3 biological replicates. (**b**) qPCR analysis of *PIN1* and *PIN2* transcript levels in wild type (WT) seedlings versus *ami-ppp1* seedlings. Graph depicts expression fold change in *PIN* gene expression in the *ami-ppp1* line relative to WT and normalized to the expression of 2 reference genes (*EIF4a* and *TUB*). Error bars depict s.e.m. from 3 biological replicates. (**c,d**) Activity of *PIN2p::GUS* in a wild type (c) and in a *ami-ppp1* (d) root meristem. (**e,f**) Whole mount immuno-labeling performed with wild type (top) and *ami-ppp1* (bottom) seedlings at 4 DAG that were probed with anti-PIN2 (e) and anti-PIN1 (f). (**g**) qPCR analysis of transcript levels of genes involved in intra- and intercellular auxin transport in wild type (WT) and *ami-ppp1* seedlings. Graph depicts expression fold change in gene expression in the *ami-ppp1* line relative to WT. Error bars depict s.e.m from 3 biological replicates. Bars: c,d = 100 μm; e,f = 20 μm.

**Figure 7:** Phenotypic analysis of *ppp1* loss-of-function lines. (**a,b**) Comparison of wild type (a) and *ami-ppp1* (b) plantlets grown on vertically orientated agar plates for 11 days. Red arrowheads indicate direction of gravity vector (**c**) Wild type (left) and *ami-ppp1* (right) plants at 35 days. (**d**) Primary root length of wild type and *ami-ppp1* seedlings at 8 DAG. Error bars represent standard deviations (n = 30 seedlings for each genotype; statistical analysis was performed using Student’s two-tailed t-test). (**e**) Orientation of primary root growth of wild type and *ami-ppp1* seedlings at 8 DAG. A total of 114 (wild type) and 118 (*ami-ppp1*) seedlings was analyzed in 3 biological repeats, and plotted as percentage of seedlings displaying <15°, <30°, <45° and >45° deviation from the vertical growth axes. Error bars indicate standard deviations. (**f,g**) Comparison of *ppp1-411* (f) and *ppp1-411 35S::PIN1* (g) primary root meristems at 9 DAG. White arrowheads depict onset of cell elongation. (**h**) Partial rescue of *ppp1-411* root elongation by *35S::PIN1*. Root lengths of wild type (WT), *35S::PIN1*, *ppp1-411* and *ppp1-411/35S::PIN1*. The latter is significantly longer compared to *ppp1-411* mutants (n ≥ 20 individuals analyzed for each genotype; statistical analysis was performed using Student’s two-tailed t-test; standard deviations are shown as error bars). Bars: a,b = 10 mm; c = 50 mm; f,g = 50 μm.

**Table 1:** Segregation of *ppp1-411* and *ppp1-476* phenotypes in the F1 generation derived from selfed heterozygote parental plants.

phenotypes observed/expected*	wild type	growth arrest	n	Χ^2^
*PPP1*/*ppp1-411*	151/139.5	35/46.5	186	3.792**
*PPP1*/*ppp1-476*	50/44.25	9/14.75	59	2.989**

^*^for a 3:1 segregation of the mutant phenotype.

^**^No significant deviation from a 3:1 segregation at p ≥ 0.05 (one degree of freedom).
